RETRACTED

# Advancements in intrusion detection: A lightweight hybrid RNN-RF model

**DOI:** 10.1371/journal.pone.0299666

**Published:** 2024-06-21

**Authors:** Nasrullah Khan, Muhammad Ismail Mohmand, Sadaqat ur Rehman, Zia Ullah, Zahid Khan, Wadii Boulila

**Affiliations:** 1 Department of Computer Science Brains Institute, Peshawar, Pakistan; 2 School of Sciences, Engineering and Environment, University of Salford, Salford, United Kingdom; 3 Robotics and Internet-of-Things Laboratory, Prince Sultan University, Riyadh, Saudi Arabia; 4 RIADI Laboratory, National School of Computer Sciences, University of Manouba, Manouba, Tunisia; Universiti Teknologi PETRONAS / University of Management and Technology, MALAYSIA

## Abstract

Computer networks face vulnerability to numerous attacks, which pose significant threats to our data security and the freedom of communication. This paper introduces a novel intrusion detection technique that diverges from traditional methods by leveraging Recurrent Neural Networks (RNNs) for both data preprocessing and feature extraction. The proposed process is based on the following steps: (1) training the data using RNNs, (2) extracting features from their hidden layers, and (3) applying various classification algorithms. This methodology offers significant advantages and greatly differs from existing intrusion detection practices. The effectiveness of our method is demonstrated through trials on the Network Security Laboratory (NSL) and Canadian Institute for Cybersecurity (CIC) 2017 datasets, where the application of RNNs for intrusion detection shows substantial practical implications. Specifically, we achieved accuracy scores of 99.6% with Decision Tree, Random Forest, and CatBoost classifiers on the NSL dataset, and 99.8% and 99.9%, respectively, on the CIC 2017 dataset. By reversing the conventional sequence of training data with RNNs and then extracting features before applying classification algorithms, our approach provides a major shift in intrusion detection methodologies. This modification in the pipeline underscores the benefits of utilizing RNNs for feature extraction and data preprocessing, meeting the critical need to safeguard data security and communication freedom against ever-evolving network threats.

## 1 Introduction

The remarkable and rapid growth of the Internet-of-Things (IoT) has increasingly drawn the attention of cybercriminals, making it more vulnerable to attacks than ever before [1]. To address these vulnerabilities, a system has been developed [2] that is independent of communication protocols, aimed at simplifying the deployment process and reducing the complexities involved [3]. In our experimental performance analysis, the proposed system demonstrated reliable and consistent effectiveness in detecting and responding to both simulated threats and real-world invasions. With an average accuracy of 93.74%, it can identify Blackhole, Distributed Denial of Service, Opportunistic Service, Sinkhole, and Workhole attacks. The average precision, recall, and F1-score of the suggested intrusion detection system are 93.71%, 93.82%, and 93.47%, respectively. The 93.21% average detection rate maintained by the cutting-edge deep learning-based intrusion detection system is enough for enhancing the security of IoT networks [4]. The objective of this research is to develop an intrusion detection model by applying various machine learning methods to specific properties identified during the modeling phase [5]. This involves using the NSL-KDD dataset to construct an Intrusion Detection System (IDS). The paper provides a concise review of multiple machine-learning techniques, including Support Vector Machines (SVM), Random Forests, and Decision Trees. These techniques aim to increase detection accuracy by analyzing attacks on the selected dataset, focusing on carefully selected key features. Additionally, the study includes a comparative analysis of these algorithms to determine the most effective approach for intrusion detection. Fig 1 shows an overview of signature-based and anomaly-based intrusion detection systems.

RETRACTED

**Fig 1:** Function of signature-based and anomaly-based IDS.

In recent years, the literature has increasingly emphasized the application of Machine Learning (ML) [6] techniques to enhance the accuracy of Intrusion Detection Systems (IDS) [7]. ML is a branch of science that seeks to replicate human learning [8]. Specifically, within the realm of Intrusion Detection Systems (IDS), ML is capable of understanding the patterns of both normal and malicious network traffic. This understanding allows it to effectively differentiate between benign and harmful activities [9]. Recent research indicates that IDS which employ ML algorithms are capable of achieving superior accuracy rates, surpassing those of conventional approaches [10, 11]. However, a common drawback of IDS is its inability to detect previously unseen attacks, particularly those classified as zero-day attacks [12, 13]. A zero-day attack happens when hackers take advantage of a system vulnerability that the developer is unaware of or has not yet been fixed [14, 15]. IDS frequently has the limitation of only being able to detect zero-day attacks and unseen attacks, despite having great accuracy in identifying known attack activity [16, 17]. Machine learning is an appropriate choice to fix the aforementioned flaw. Drawing inspiration from the comprehensive analysis [18], which explores various machine learning techniques such as decision tree (DT), random forest (RF), support vector machine (SVM), naive Bayes (NB), artificial neural network (ANN) [19, 20], and deep neural network (DNN) [21] for simulating zero-day attacks, our study aims to build upon and extend their findings. We introduce novel contributions in the realm of intrusion detection systems as follows:

- We make a significant contribution by using RNNs for feature extraction before any feature selection, which has the potential to identify intrusion patterns that may not be explicitly defined in traditional handcrafted features.
- Selection of numerous datasets for the evaluation, including the NSL-KDD and the CIC-IDS2017.
- Our approach’s ability to maintain or improve accuracy while reducing processing time demonstrates practical value for deployment in resource-constrained environments.
- We also employed various feature selection methods and determined the most effective feature selection method.

RETRACTED

Given the limitations inherent in traditional signature-based methods and the challenges posed by false positives in anomaly-based detection, our research investigates a pivotal question: Can the accuracy and efficiency of intrusion detection systems, particularly in resource-constrained environments, be significantly enhanced by employing RNNs for feature extraction before feature selection? This approach aims to unveil complex intrusion patterns that elude detection by conventional handcrafted features, potentially revolutionizing how systems identify and respond to security threats.

The paper is organized as follows: The Background Study section reviews relevant background work, while Proposed System section introduces our proposed system and the machine learning models employed. Model evaluations and the discussion of results are presented next, leading to the Conclusion and Future Work section, which offers a conclusion that summarizes our findings and suggests directions for future research.

## 2 Background study

Over the past decade, there has been considerable exploration into the integration of ML into IDS [22, 23]. A review by Md.Alamgir at [24] employing various ensemble techniques shows that the suggested strategy utilizing the Random Forest technique beats previous strategies in terms of accuracy and FPR, usually above 99% with superior assessment metrics. The authors in [25] used an auto-encoder as a label. A deep-learning classification model [26] was trained on the KDD data set, which achieved an average accuracy of 85%.

In the study [27], A new architecture for deep neural networks that can train flexible and robust models for intrusion detection is established by merging the multichannel feature learning stage of the unsupervised setting with the supervised set of cross-channel feature correlation [28]. Specifically, in the unsupervised stage [29], two autoencoders are trained during the normal and attack procedures. The top layer of the decoder of these autoencoders revamps tests as a contribution to a similar space, permitting them to be utilized to create two different component vectors, allowing each organization stream to be addressed as a multichannel test [30, 31]. During the supervision phase, multichannel parameter convolution is utilized to understand how one channel affects the others [32, 33]. Since the examples come from two unmistakable distributions (typical and assault stream), the ordinary models should be more pertinent to an assault than the portrayal remade utilizing a standard autoencoder, and vice versa [34]. Their expected dependency can improve the geographical removal of flows. The proposed neural network design can improve prediction accuracy in the following scenarios. On three benchmark data sets, they examined rival intrusion detection architectures [35, 36]. In the review [37], the PSO-Xgboost model is introduced because it outperforms competing models like Xgboost, Irregular Backwoods, Stowing, and Adaboost regarding overall order precision.

RETRACTED

Imran *et. al*. [38], proposed a hybrid feature selection method based on the random forest model and Pearson correlation coefficient. For the machine learning (ML) model, the decision tree, AdaBoost, and K-nearest neighbor are trained and tested on the TON-IoT dataset. The dataset is fresh and includes features and attack kinds that are new and current [39]. Multilayer perceptrons (MLPs) and long short-term memory are trained and tested for deep learning [40, 41]. The criteria used for evaluation include recall, accuracy, and precision. Recent research has demonstrated that IDS with machine learning models can achieve high accuracy rates exceeding 90% [42, 43]. As a result, some studies have shifted their focus to comparative analyses, where numerous models are applied and assessed using varied datasets. Shema and Saad in 2023 [44] propose an innovative strategy employing a combination of deep learning and three-level algorithms to detect threats in IoT networks quickly and accurately. The suggested method is evaluated using the Bot-IoT dataset, and the outcomes demonstrate notable gains in detection performance over current techniques [45, 46]. The suggested method is a promising addition to the field of IoT security since it can be expanded to improve the security of additional IoT applications [47–53].

RETRACTED

The paper [54] proposed a malware analysis and detection with machine learning algorithms to compute the difference in correlation symmetry (Naive Byes, SVM, J48, RF, and with the proposed approach) integrals could be used to detect harmful traffic on computer systems, thereby improving the security of computer networks. The findings demonstrated that DT (99%), CNN (98.76%), and SVM (96.41%) performed well in terms of detection accuracy when compared to other classifiers. In the paper [76], the authors proposed using adversarial machine learning for malware and intrusion detection scenarios. We concluded that, while their applicability in intrusion scenarios was not tested, a wide range of attacks were evaluated and shown to be successful in malware and intrusion detection. IDS’s primary goal is to identify intrusion activity by looking for a suspicious trend in the events that are being recorded. The normal and attack user datasets were first gathered via the Internet of Things and fed into the system for training.

In light of this, a brand-new Bear Smell-based Random Forest (BSbRF) was created to detect intrusions accurately [55] by keeping an eye on their behavior about their threshold value. In the publication [56], the proposed traffic anomaly detection model is BAT. Bidirectional Long Short-Term Memory (BLSTM) and the attention mechanism are combined in the BAT model. The network flow vector comprised of packet vectors produced by the BLSTM model is screened using an attention mechanism to extract the essential characteristics needed to classify network traffic [57, 58]. in addition, a network intrusion detection technique combines deep hierarchical networks and hybrid sampling. First, we lower the noise samples in the majority category using one-side selection (OSS). Then, we utilize the Synthetic Minority Over-sampling Technique (SMOTE) [59] to augment the minority samples.

In [60], the authors proposed applying AI (Machine Learning) approaches for intrusion detection. They utilized the KDD dataset from the UCI archive. They executed different administered or supervised models to adjust non-arrangement algorithms for better execution. They have accomplished excellent outcomes in this work. To identify an adversary’s attempts to inject undesired data into an IoT network, the authors in a study [61] created a lightweight attack detection technique based on supervised machine learning-based support vector machines. The reenactment results showed that the recommended SVM-based classifier worked as far as grouping exactness and recognition time when empowered by a blend of a few complex elements.

RETRACTED

The proposed work [62] outlined common IoT protocols and the vulnerabilities that go along with them. After that, a cyber-vulnerability assessment was conducted, which described how machine learning might be utilized to reduce these risks. Using merely 1% of the NSL-KDD KDDTrain+dataset for training, the intrusion detection approach described in the paper [63] achieved 92.34% accuracy for the KDD-Test and 85.75% accuracy for the KDD-Test-21. The review [64] proposed an organization interruption recognition method in light of a convolutional brain network-IDS (CNN-IDS). First, repetitive and unnecessary qualities in network traffic information are eliminated using different dimensionality decrease techniques. KDD-CUP99 dataset was used [65]. The results of AC, FAR, and timeliness reveal that the CNN–IDS model outperforms existing methods. In [66], a profound learning-based interruption recognition framework (IDS), because of feed-forward deep brain organizations (FFDNNs) and a channel-based highlight determination approach, was created. NSL-KDD dataset on the test set made a precision of 86.62%.

The authors in [67], proposed AI-SIEM system using various artificial neural network techniques, such as CNN, LSTM, and FCNN, together with event profiling for data preparation. The approach helped security analysts react quickly to cyber threats by focusing on differentiating between true positive and false positive signals. The authors of this work conducted all of the experiments using two real-world datasets and two benchmark datasets, NSLKDD and CICIDS2017. Five traditional machine-learning techniques (SVM, k-NN, RF, NB, and DT) were used to assess the performance comparison with current methodologies. As a result, the experimental findings of this work guarantee the applicability of our suggested techniques as learning-based models for network intrusion detection and demonstrate that while. Table 1 summarises the whole review.

**Table 1:** Literature review comprising main studies.

Study	Methodology	Datasets	Key finding
Md.Alamgir [6]	ensemble techniques	various datasets	99 accuracy using RF
Yang Y [7]	auto-encoder	KDD	85 accuracy using deep learning
*Andresini* [8]	Un-sv + sv DNN	unspecified	better accuracy using benchmark datasets
Jiang H [9]	PSO-Xgboost	NSL-KDD	Outperformed competing models
*Imran* [10]	hybrid feature selection	TON-IoT	achieve high accuracy rates exceeding 90
*Shema* [11]	DL and three-level algorithms	Bot-IoT	improve the security of IoT applications
*Martins* [13]	adversarial machine learning	various datasets	successful in malware and intrusion
*Alalayah* [14]	Bear Smell-based RF	IoT-based	detect intrusions accurately
*Su T* [15]	BLSTM	benchmark	accuracy is largely improved
*Jiang K* [16]	hybrid sampling deep hierarchical network	NSL-KDD UNSW-NB15	accuracy can achieve 83 and 77
*Nagaraja* [17]	Machine Learning approaches	KDD	99% accuracy
*Karatas* [61]	supervised ML-based	CIC-IDS2018	Adaboost is the most successful
*Zolanvari* [19]	outline common IoT protocol	Built dataset	New types of attack such as backdoor, command injection
*Yu Y*, [20]	Few-Shot Learning (FSL)	NSL-KDD	92.34% accuracy
*Xiao*, [21]	CNN-IDS	KDD-CUP99	convert the original traffic vector into an image format
*Kasongo* [22]	feed-forward deep brain and a channel-based approach	NSL-KDD	made a precision of 86.62%
*Lee J*, [23]	AI-SIEM system	NSLKDD CICIDS2017)	capable of being employed as learning-based models)

RETRACTED

## 3 Proposed system

In this part, we provide a cutting-edge intrusion detection algorithm that challenges the standard method, as shown in Fig 2. RNNs are used to train the data in our method. Random Forest is used to select features, and finally, a variety of classifiers, including Decision Trees, Random Forest, and Boosting algorithms (AdaBoost, boost, and XGBoost), are used. To assess the efficacy of this novel technique, it is applied to the NSL-KDD and CIC-2017 datasets. We execute crucial data pretreatment procedures to ensure the datasets are appropriate for analysis before applying our new technique. This comprises categorical feature encoding, resolving missing values, and data cleaning.

**Fig 2:** Proposed solution of IDS.

To improve the model’s comprehension of complicated network intrusion scenarios, we train the data with RNNs to develop robust data representations. We go on to feature extraction after RNN data training. In this stage, we use the RNNs’ learned information to extract pertinent characteristics from the data. This ensures that the model’s knowledge of the subtleties and underlying patterns in the dataset informs the selection of the features. Using Random Forest as the feature selection method, we further improve the feature set after feature extraction. By doing feature selection after feature extraction, our methodology varies dramatically from traditional approaches. As a result, the model may direct the selection procedure using its learned data representations, potentially revealing non-trivial aspects that are significant to the context.

After classification, in terms of precision, recall, and F1 score, authors perform performance measures. Finally, the authors compare the work with existing ones. We use a variety of classifiers to perform intrusion detection using the chosen characteristics. Decision Trees (DT), Random Forest (RF), AdaBoost, Catboost, and XGBoost are some of the classifiers in this group. To test each classifier’s capacity to discriminate between legitimate and malicious network activity, a dataset containing the chosen attributes is used to train each classifier. Our methodology is also designed to offer fast response times for real-time intrusion detection applications, ensuring timely decision-making.

RETRACTED

We use XG Boost, Decision Tree, Random Forest, and Catboost classifiers. XG Boost is considered one of the best machine learning algorithms because of cache optimization, auto pruning, parallelization, out-of-memory computation, regularization, and missing value handling. The five classifiers are used on the following datasets. The goal is to learn about data integrity and improve data prediction accuracy.

A flow chart of the proposed methodology is presented in Fig 3.

**Fig 3:** Flow chart of the proposed methodology.

### 3.1 Dataset

The lack of accessible datasets is one of the main challenges facing researchers of intrusion detection systems (IDS). This is because many organizations are reluctant to share their network traffic data due to concerns about privacy and security. Nonetheless, having a reliable dataset is essential for building an anomaly-based IDS and assessing its effectiveness. As a result, numerous datasets have been created by various organizations for research purposes. This section will introduce the datasets that were utilized in our research.

### 3.2 NSL-KDD dataset

NSL-KDD is a data collection proposed to address some of the shortcomings of the KDD’99 data set. The NSL-KDD train and test sets have a reasonable amount of recordings. This benefit makes it feasible to execute the trials on the entire collection rather than a small subset at random. The proportion of records chosen from each difficulty level group is inversely proportional to the proportion of records in the original KDD dataset. As a result, various machine learning approaches have a greater variety of categorization rates. This method improves the accuracy of assessing various learning strategies.

### 3.3 2017 CIC-IDS dataset

The 2017 CIC-IDS Dataset dataset is a well-known and widely used dataset that has gained popularity in recent years. It was developed in 2017 by the Canadian Institute for Cybersecurity (CIC) and offers a diverse range of operating systems, protocols, and attack types. The dataset is especially valuable as it covers a wide range of contemporary operating systems, including Windows, Mac OS, and Ubuntu, and was created in a comprehensive network environment with various components such as modems, firewalls, switches, and routers. Using protocols including HTTP, HTTPS, FTP, SHH, and other email protocols, the behaviour of 25 users was mimicked to provide benign traffic for the dataset. The most common assaults in 2016—brute force attacks, denial of service attacks, distributed denial of service attacks, intrusion attacks, Heartbleed attacks, botnet attacks, and port scan attacks—were recreated. Once the dataset was complete, it was made publicly available in CSV file format on the University of New Brunswick website [68]. The major drawback of the dataset is the high class imbalance issue, with over 70% of the traffic being benign and only a few attacks constituting less than 1% of it [69].

RETRACTED

### 3.4 Data pre-processing

Data wrangling, also known as data cleaning, involves preparing data by removing unwanted values, null items, and other inconsistencies [70]. This process is a crucial stage in data mining, aimed at ensuring the data is clean for accurate analysis [71]. During this step, the authors apply preprocessing techniques to examine the data, removing any invalid or missing values, as well as duplicates. By eliminating absent or empty attributes and duplicates, the authors ensure the data is well-prepared for further analysis. This complex and essential step advances the clarity and precision of data analysis.

### 3.5 Data visualization

The graphic structure’s data address it just through visual information on the information that it is feasible to choose [72]. Close perception information and Matplotlib, information depiction information is accessible. In this section, the authors exhibit our data set visually. It is enough to interpret the data better and make algorithm decisions. Figs 4 and 5 depict attacks in a graphical style that shows all intrusions. Fig 4 depicts attacks in a graphical style that shows all intrusions. The CIC-IDS2017 dataset comprises five categories, with the first one being benign (2096134), followed by DoS Hulk (172846), DDoS (128016), PortScan (90819), and finally DoS GoldenEye (10286). In the NSL-KDD dataset, the first one is normal (67343), followed by Dos (45929), Probe (11656), r2l (995), and u2r(52). Now, we use the above actual intrusion for classification and prediction by our understudy machine learning models. It is our target class for a model. The next step is featuring scaling to remove overfitting from the data set to make the data have a normal form. That can help in model training for best learning.

**Fig 4:** Depicts attacks on CIC-IDS2017.

**Fig 5:** Depicts attacks on NSL-KDD.

All the machine learning algorithms use input data [73]. This input data set has structural columns as features [74]. All calculations need the utilization of information highlights with specific characters to work appropriately. Providing an input data collection compatible with the machine learning model specifications is the primary aim of feature engineering. Accordingly, the authors start by changing overall downright properties into mathematical qualities. Second, to work on the AI (Machine Learning) model exhibition. Authors use the feature scaling technique to balance the independent variables in the dataset over a specific range. It handles the value, magnitude, value, or unit of height variation during data processing. Without feature scaling, regardless of the unit of value, the machine learning algorithm will give less importance to smaller values and more importance to higher values. For feature scaling implementation, two optimal approaches given below are used.

RETRACTED

### 3.6 Standardization

As a first approach, standardization is utilized, and it is the method involved with deducting your information by the process for all perceptions and partitioning the outcome by the standard deviation, followed by scaling your perceptions [75]. In AI, the accompanying recipe is utilized for normalization. It is a very effective strategy for rescaling the information to create a dispersion with a mean of nothing and a change of one.

$$\begin{array}{c} Xnew=\frac{x_{i}-Xmean}{standardDeviation} \end{array}$$ (1)

### 3.7 Normalization

Normalization includes deducting your perception from the base, everything being equal, separating by the most significant number of perceptions, and afterward scaling the component. This approach rescales elements or perceptions with a circulation esteem between 0 and 1.

$$\begin{array}{c} Xnew=\frac{x_{i}-min\left(x\right)}{man(x)-min(x)} \end{array}$$ (2)

The authors apply a typical scalar feature scaling approach for feature scaling in our proposed study. Since it is the most effective method for scaling different label features in supervised learning models. Machine learning algorithms utilize artificial intelligence to take and refine data without being expressly modified. AI is worried about the advancement of PC frameworks that can acknowledge and gain from data [76]. Prior knowledge is used to supervise classification algorithms that employ categorical data sets for classification and prediction tasks. Also, the authors used the model optimization technique to improve model performance. The following are the results of the algorithms used in this research study.

## 4 Machine learning models

Machine learning (ML) and its potential applications in numerous fields have drawn increasing attention in recent years [77]. The ability of ML models to predict or categorize data is very strong. In Intrusion Detection Systems (IDS), ML is used to distinguish between legitimate and malicious network traffic. Some of the most popular ML models in IDS are briefly described in this section.

RETRACTED

### 4.1 Recurrent Neural Network (RNNs)

Recurrent neural networks (RNNs) are a type of artificial neural network designed for processing data sequences. The fundamental structure of an RNN involves the following components. Input Sequence: An RNN receives a data sequence as input. This sequence can be of various lengths and represent time series data, natural language phrases, or any other sequential data. let *X*_*t*_ be the input at time step t,*W*_*hx*_ is the weight matrix connecting the hidden state to the input. *H*_*t*−1_ is the previous hidden state, *W*_*hh*_ is the weight of the matrix for recurrent connections *H*_*t*_ be the hidden state at the time step t. Then, the combination of the hidden state can be expressed as

$$\begin{array}{c} X_{t}=activation\left(W_{hx}.x_{t}\right)+W_{hh}.H_{t-}1 \end{array}$$ (3)

$$\begin{array}{cc} & \left(x\right)=\frac{1}{1+e^{z}} \end{array}$$ (4)

Rectified Linear unit (ReLU): ReLU(x) = max (0, x) These functions are applied element-wise to the outputs of matrix multiplication.

### 4.2 Random Forest

An RF is a troupe learning strategy that frames an enormous gathering of free-D-tree and results in the method of the name forecasts of the multitude of trees. This technique has more prominent registering costs yet decreases overfitting of the information, which happens when a model adjusts too stringently to a specific arrangement of information, having unfortunate capacities for speculation. An RF classifier depends on a group of RF classifiers H(x|*θ*1………h(x|) based on a classification tree with parameter *θk* is randomly selected the random vector model *θ* For the last classification, f(x), which is used to combine the classifiers {h_*x*_(*x*)} *respectively*.

### 4.3 Decision Tree

One of the fundamental Supervised ML techniques, DT applies a series of decisions (rules) to characterize the dataset and perform regression on it. It has a predefined objective variable and is upheld by a leaf hub. A portion of the leaf hubs is wiped out from the D-tree to avoid Overfitting. Entropy and data gain ought to be determined for the D-tree, so how entropy ought to be selected is given in Eq 5.

$$\begin{array}{c} E\left(S\right)=\sum_{x\propto X}^{n}-p\left(a\right)E\left(a\right) \end{array}$$ (5)

S is a dataset, X is a collection of classes inside S, and p is a ratio of the number of entries within class X. Eq 6 thus illustrates the calculation of knowledge gain

$$\begin{array}{c} Gain\left(A,S\right)=E\left(S\right)-\sum_{x\propto T}^{n}-p\left(a\right)E\left(a\right) \end{array}$$ (6)

Where subsets are created from the dataset S as a T.

RETRACTED

### 4.4 AdaBoost classifier

Machine learning is also used as a classification algorithm that uses labelled data. It is the same as XGBoost but utilizes only two levels of the decision tree. It works on probability. This approach is used to represent the classification performance of machine learning. Authors may acquire an improved understanding of the classification model’s accuracy and the sort of error generated by computing the confusion matrix. It is used to measure classification accuracy and categorize accurate and predicted labels. They present a visual representation of the classifier’s performance.

### 4.5 XGBoost classifier

XgBoost is another machine learning algorithm that is analyzed in this research. XGBoost is a widely used machine learning technique, and it’s gotten a lot of attention recently since it’s speedy, especially when working with enormous data sets. The accuracy, speed, and size of XGBoost have matured into models for data science challenges. As a result, it is critical to achieve high levels of accuracy and execution speed. XGBoost Classifier is 100 times quicker than previous algorithms and similar to a tree. It functions admirably with enormous informational indexes [78].

### 4.6 CatBoost

Below are the results and performance obtained through the CatBoost classifier, a gradient-boosting algorithm working on a tree. It is compelling and widely used for future forecasting for probability. This model can perform at high performance without a GPU. This means this model is more likely to perform than other boosting models.

## 5 Model evaluation

This section includes results from classifiers and an overview of our proposed model. For the intended study, the authors chose the Python programming language. This programming language is simple and can be customizable. The language’s best-desired position is to employ minimal code and implicit libraries with explicit practicality. In the Jupyter Notebook, authors use Python. The Jupyter Notebook is a fast, open-source editor. The authors selected the CIC-IDS2017 and NSL-KDD, containing information about intrusion data in the latest version. The authors utilise the most recent dataset to categorize the current level of incursion. The total number of rows and columns in the CIC-IDS2017 dataset is 2830743 and 79, respectively. In NSL-KDD, there are (125973) rows and 42 columns. The authors used essential Python libraries to read and write data for further processing. Each of these libraries has its capabilities for doing various tasks.

### 5.1 Feature selection CIC-IDS

A crucial stage in creating a machine learning model is feature selection. By focusing on the features that have the greatest impact on the target variable, feature selection reduces the complexity of the dataset. By doing so, it can help in improving the accuracy of the model, reducing the training time, and avoiding overfitting. In paper [79], the feature selection problem was turned into an optimization problem using the Hybrid Ant-Bee Colony Optimisation (HABCO) technique. In [80], the fusion of the Statistical Importance-based feature selection technique is used. The CIC-IDS2017 dataset is used in its entirety and contains about 80 features. Training the model without any feature selection will take time. In addition, some features could introduce noise and decrease the model’s accuracy. Following RNN-based pre-processing, we use Random Forest as a feature selection technique. This hybrid method takes advantage of RNNs’ temporal modeling skills as well as Random Forest’s capacity to rank and choose the most important characteristics.

RETRACTED

### 5.2 Performance evaluation

The confusion matrix represents the total number of actual and expected classification labels. It combines True Negative (TN), True Positive (TP), False Negative (FN), and False Positive (FP) values to produce actual and anticipated labels. We calculate the model’s classification and prediction accuracy based on these values:

1. True-Negative: the number of accurate predictions that a case has received.

2. True-Positive: the percentage of accurate predictions indicating a positive outcome

3. False-Positive: the number of inaccurate predictions that show a positive instance.

4. False-Negative: the quantity of false forecasts that lead to a negative event.

The labels of the confusion matrix are false negative, true positive, true negative, and false positive. Furthermore, using the aforementioned confusion matrix, we assess the performance of the suggested model.

### 5.3 Performance measure of CIC-IDS

In this step, the reliability of the models is achieved. Table 2 displays the accuracy score for each model, indicating that all models achieved an accuracy score higher than 99%. Moreover, the standard deviation of each model’s accuracy is minimal, demonstrating that, using the CIC-IDS2017 dataset, the accuracy of each model is quite consistent. On the other hand, the CatBoost model performed the best, achieving an accuracy of 99.99%, which is a significant accomplishment. Table 3 compare the accuracy of the proposed approach with different models.

**Table 2:** Accuracy results on the CIC-IDS2017 dataset.

Model	Accuracy	F1-Score	Precision	Recall
*DecisionTree*	0.9987	1.00	1.00	1.00
height *RandomForest*	0.9989	1.00	1.00	1.00
*XGBoost*	0.9716	0.94	0.97	0.92
*AdaBoost*	0.9958	0.99	0.99	0.99
*CatBoost*	0.9993	1.00	1.00	1.00

RETRACTED

**Table 3:** Using the CIC dataset, accuracy comparison with other literature.

Model	Proposed Model	Tuan-Hong Chua [22]	Kostas [30]
*DecisionTree*	1.00	0.995	0.95
*RandomForest*	1.00	0.996	0.94
*XGBoost*	0.9716	-	-
*AdaBoost*	0.9958	-	-
*CatBoos*	0.9993	-	-

We assessed the accuracy of the classification outcomes and predictive findings using the confusion matrix. Figs 6–10 display the confusion matrices and classification results for Decision Tree, Random Forest, Naïve Bayes, XGBoost, AdaBoost, and CatBoost.

**Fig 6:** Confusion matrix of DT.

**Fig 7:** Confusion matrix of RF.

**Fig 8:** Confusion matrix of XGboost.

**Fig 9:** Confusuion matrix of AdaBoost.

**Fig 10:** Confusion matrix of CataBoost.

### 5.4 Model evaluation NSL-KDD

In this work, we employed a variety of machine learning methods, including Decision Trees (DT), Random Forest (RF), XGBoost, CatBoost, and AdaBoost. We achieved an outstanding 99% accuracy on the NSL dataset for intrusion detection. This exceptional precision underscores the effectiveness of our strategy in enhancing cybersecurity measures. Our findings highlight the considerable potential of these algorithms for intrusion detection tasks on the NSL dataset as shown in Table 4, setting the stage for future efforts in cybersecurity.

**Table 4:** The accuracy result on NSL-KDD dataset.

Model	Accuracy	F1-Score	Precision	Recall
*DecisionTree*	0.9965	1.00	1.00	1.00
*RandomForest*	0.9969	1.00	1.00	1.00
*XGBoost*	0.9976	1.00	1.00	1.00
*AdaBoost*	0.9846	0.98	0.97	0.98
*CatBoost*	0.9960	0.99	1.00	0.99

Confusion matrix and classification results of the NSL-KDD dataset are displayed in Figs 11–15. Figures expound the confusion matrix for all model execution recognizable proof. On the NSL-KDD dataset, the results of DT, RF, XGBoost, and CatBoost are consistent with those obtained on the CIC-IDS2017 datasets. However, the XGBoost algorithm achieved an excellent accuracy of 99.97% on the NSL dataset, demonstrating its extraordinary ability in intrusion detection. Table 5 shows the comparison analysis of the proposed model with other models present in the literature.

**Fig 11:** Confusion matrix of DT.

**Fig 12:** Confusion matrix of RF.

**Fig 13:** Confusion matrix of XGboost.

**Fig 14:** Confusuion matrix of AdaBoost.

**Fig 15:** Confusuion matrix of CataBoost.

**Table 5:** Using the NSL dataset to compare accuracy to other research.

Model	Proposed Model	Tuan-Hong Chua [22]	Kostas [30]
*DecisionTree*	1.00	0.9994	-
*RandomForest*	1.00	0.9994	-
*XGBoost*	1.00	-	-
*AdaBoost*	0.98	-	-
*CatBoost*	1.00	-	-

Additionally our approach of training the model before classification not only enhances accuracy but also optimizes the computational efficiency of intrusion detection. model performance comparisons on the training and testing dataset are shown in Figs 16–18. In Fig 16 our approach of training the model before feature selection leads to significantly better results compared to the traditional approach, Furthermore, relative to their recall scores, both models have inferior precision scores on the benign class of the *NSLKDD* and CIC-2017 datasets. According to Figs 17 and 18, AdaBoost are the most time-consuming models for training, while DT, RF, CatBoost, and XGboost remain the most efficient

RETRACTED

**Fig 16:** Models’ F1-score and accuracy on the NSL-KDD dataset and CIC207.

**Fig 17:** CIC-2017 dataset training period.

**Fig 18:** NSLKDD dataset training period.

The time complexity of each model is a significant component that impacts the training duration in addition to the previously listed factors. Each model has its unique algorithmic structure and computational requirements, which result in different time complexities. For instance, AdaBoost typically requires more computations and memory compared to DT, RF, and Catboost due to their complex algorithms. Consequently, AdaBoost is more time-consuming for training, whereas DT, RF, NB, XGboost, and CatBoost are less demanding and, therefore, more efficient in terms of training time.

## 6 Results and discussion

In our method, we present the outcomes of our innovative approach, which entails training the data using recurrent neural networks (RNNs) before feature selection with random forests (RF), followed by classification using different classifiers, including decision trees (DT), random forests (RF), and boosting algorithms (AdaBoost and XGBoost).

In this study, we introduce a novel approach for intrusion detection that initially employs Recurrent Neural Networks (RNNs) for data training, followed by Random Forest for feature selection, and various classifiers for the classification process. The experimental results on the NSL-KDD and CIC-2017 datasets as shown in Tables 6 and 7 illustrate the effectiveness of our strategy in achieving high accuracy while reducing training time. Our method combines the benefits of enhanced accuracy and computational efficiency, making it a practical choice for real-world intrusion detection systems. Our research challenges the traditional sequence of operations and highlights the importance of data-driven feature selection following model training, thereby advancing the field of intrusion detection. We believe our approach opens new avenues for efficient and accurate intrusion detection and warrants further investigation in practical application settings. Our focus lies on the unique aspect of our strategy—utilizing Recurrent Neural Networks (RNNs) for initial model training before employing Random Forest for feature selection. The aim of this hybrid technique is to boost the model’s performance.

RETRACTED

**Table 6:** NSL-KDD dataset results.

Model	Accuracy	F1-Score	Precision	Recall	Training time in (s)
*RNN* + *RF* + *DT*	0.9965	1.00	1.00	1.00	0.32
*RNN* + *RF* + *RF*	0.9969	1.00	1.00	1.00	1.13
*RNN* + *RF* + *XGboost*	0.9976	1.00	1.00	1.00	1.25
*RNN* + *RF* + *Adaboost*	0.9846	0.98	0.97	0.98	3.95
*RNN* + *RF* + *Catboost*	0.9960	0.99	1.00	0.99	0.95

**Table 7:** CIC-IDS2017 result.

Model	Accuracy	F1-Score	Precision	Recall	Training time in (s)
*RNN* + *RF* + *DT*	0.9987	1.00	1.00	1.00	46.39
*RNN* + *RF* + *RF*	0.9989	1.00	1.00	1.00	80.74
*RNN* + *RF* + *RF*	0.9716	0.94	0.97	0.92	81.22
*RNN* + *RF* + *Adaboost*	0.9958	0.99	0.99	0.99	361.90
*RNN* + *RF* + *Catboost*	0.9993	1.00	1.00	1.00	19.09

In this work, we conducted two tests: one using the datasets from CIC and the other using the dataset from NSL-KDD. Interestingly, the outcomes of both experiments were the same. Our research indicates that XGBoost and CatBoost are the most suitable models for environments where the system’s infrastructure is regularly updated and the cost of cyberattacks is significant. This is because XGBoost and CatBoost balance prediction time and resistance to overfitting effectively. Conversely, if a system’s infrastructure is not frequently updated and is less vulnerable to large-scale attacks, Decision Trees (DT) and Random Forest (RF) are preferable options. DT provides the best accuracy on the training dataset in both studies, proving to be very effective in training and classifying new samples.

## 7 Conclusion and future work

In this study, we aimed to address the critical issue of reaction time efficiency while advancing the accuracy of intrusion detection. Our approach involves a two-step process: initial model training using Recurrent Neural Networks (RNNs), followed by feature selection with Random Forest, which has demonstrated outstanding results on two well-known datasets, NSL and CIC-2017. For our experiments, we selected these datasets to test five machine learning models: XGBoost, CatBoost, Random Forest, Decision Tree, and AdaBoost. We standardized the data before applying the suggested supervised learning algorithms to generate classification and prediction results.

Our method stands out because it strikes a balance between accuracy and reaction time, offering a practical solution to the intricate issue of intrusion detection. We employ Recurrent Neural Networks (RNNs) for initial model training, enhancing the system’s resilience and adaptability. Following this, Random Forest is utilized for feature selection, ensuring the model’s effectiveness. Our findings carry significant implications for the cybersecurity industry, marking a considerable step forward in bolstering an organization’s security posture. This enables quicker and more accurate threat assessments, which we believe will greatly enhance incident response capabilities in real-world cyber environments. In our view, the combination of high accuracy and rapid reaction times is crucial for improving incident response in actual cybersecurity settings.

RETRACTED

Although our method has shown remarkable promise, we recognize several limitations, including the necessity for further testing across diverse datasets and the risk of over-fitting specific datasets. Future research should explore how effectively our method can scale to accommodate larger datasets, more complex infiltration scenarios, and evolving cybersecurity threats. In conclusion, our research marks a significant advancement in the field of intrusion detection. We have demonstrated that achieving high accuracy does not have to compromise reaction time effectiveness. Our innovative approach paves the way for enhancing the practical efficacy of intrusion detection systems. Our findings offer valuable insights for developing more efficient and reliable cybersecurity solutions as the cybersecurity landscape continues to evolve.

NSL-KDD and CIC-2017 were the only datasets utilized in the study. While these datasets are widely recognized benchmarks in intrusion detection research, they may not fully capture the diversity of real-world situations and network configurations. Employing a broader range of datasets could enhance understanding of our strategy’s generalizability. Additionally, class imbalance, a common issue in intrusion detection datasets where some classes of intrusions are significantly less common than others, can lead to model bias towards the majority class, negatively impacting the performance of minority classes. Improving the model’s resilience by addressing this imbalance through methods such as oversampling, undersampling, or employing sophisticated algorithms designed specifically for imbalanced data could mitigate this issue.
